The article "Recent development in clinical applications of PD-1 and PD-L1 antibodies for cancer immunotherapy" was published in 2017. Journal: J Hematol Oncol.

# Recent development in clinical applications of PD-1 and PD-L1 antibodies for cancer immunotherapy

**DOI:** 10.1186/s13045-017-0541-9

**Published:** 2017-12-01

**Authors:** Bingshan Liu, Yongping Song, Delong Liu

**Affiliations:** 1 School of Basic Medical Sciences and the Affiliated Cancer Hospital of Zhengzhou University, Zhengzhou, China; 2 Henan Cancer Hospital and the Affiliated Cancer Hospital of Zhengzhou University, 127 Dongming Road, Zhengzhou, 450008 China

## Abstract

Antibodies against programmed death (PD) pathway are revolutionizing cancer immunotherapy. Currently five antibodies against PD-1/PD-L1 have been approved. The clinical use of these antibodies is rapidly expanding. Incorporation of PD antibodies into chemotherapy regimens is in active clinical investigations. The combination of pembrolizumab with carboplatin and pemetrexed has been approved for the first line therapy of metastatic non-squamous non-small cell lung cancer. Combination of PD-1/PD-L1 antibodies with small molecule inhibitors such as tyrosine kinase inhibitors and IDO inhibitors are in active clinical trials. This review summarized recent development in clinical trials of PD-1 and PD-L1 antibodies for cancer immunotherapy.

## Background

Targeted therapies for cancer with small molecules and monoclonal antibodies (MoAb) have led to significant improvement in the long-term survival of multiple malignancies [1–11]. The discovery of programmed death-1 (PD-1) and the ligand 1 (PD-L1) has opened the door to the modern era of cancer immunotherapy [12, 13]. It is well known now that many tumor cells are able to upregulate the expression of PD-L1 which leads to anergy of cytotoxic T cells upon PD-1 binding to the ligand. Blocking the PD-1 pathway using monoclonal antibodies against PD-1 or PD-L1 can therefore revamp the immune response against tumor cells [14]. The development of MoAbs against PD-1 and PD-L1 has led to the fast and fundamental paradigm shift in cancer therapy [15]. The anti-PD drugs are the new form of tumor-site immune modulation therapy through resetting immune reservoir in the tumor microenvironment [16, 17]. This is fundamentally different from the conventional chemotherapy and radiation that mainly target cancer cells themselves.

PD-L1 expression on the tumor cells and immune cells have become biomarkers that can assist clinical decisions in the choice of treatment strategies [18, 19]. Biomarker assays for PD-L1 are playing bigger roles and are being routinely done nowadays. However, PD-L1 assays can be highly variable, which makes it a clinical challenge to employ the results. In this review, we summarized latest clinical development of PD antibodies and immunohistochemistry (IHC) assays for PD-L1 biomarker expression in clinical practice.

The article "Recent development in clinical applications of PD-1 and PD-L1 antibodies for cancer immunotherapy" was published in 2017. Journal: J Hematol Oncol.

## New development in clinical applications of PD-1 and PD-L1 antibodies

The US Food and Drug Administration (FDA) has approved 5 immune checkpoint blockers in 11 types of advanced malignancies (Table 1).

**Table 1:** Clinical applications of PD-1 and PD-L1 antibodies

Antibodies	Dosages^a^	Indications^b^
Pembrolizumab	200 mg over 60 min q3 weeks	Melanoma, NSCLC, HNSCC, urothelial carcinoma, Hodgkin’s lymphoma, MSI-high cancer, gastric cancer
	200 mg over 60 min q3 weeks carboplatin/pemetrexed	First line combination therapy for metastatic non-squamous NSCLC
Nivolumab	240 mg over 60 min q2 weeks	Melanoma, NSCLC, renal cell carcinoma, urothelial carcinoma, MSI-high /dMMR CRC, HCC
	3 mg/kg over 60 min q2 weeks	Hodgkin’s lymphoma, HNSCC
Atezolizumab	1200 mg over 60 min q3 weeks	Urothelial carcinoma, NSCLC
Durvalumab	10 mg/kg over 60 min q2 weeks	Urothelial carcinoma
Avelumab	10 mg/kg over 60 min q2 weeks	Merkel cell carcinoma, urothelial carcinoma

Abbreviations: *NSCLC* non-small cell lung cancer, *HNSCC* head/neck squamous cell carcinoma, *MSI* microsatellite instability; *dMMR* deficient mismatch repair gene, *CRC* colorectal cancer, *HCC* hepatocellular carcinoma, *min* minute, *q3w* every 3 weeks

^a^Ffor pediatric dosing and for combination dosage and schedules, please refer to full prescribing information for each individual agent

^b^For exact indications, please refer to full prescribing information for each individual agent

Nivolumab has FDA approved indications for treatment of eight types of advanced malignancies. These malignancies include melanoma, NSCLC (non-small cell lung cancer), classical Hodgkin lymphoma, HNSCC (squamous cell carcinoma of the head and neck), renal cell carcinoma, urothelial carcinoma, hepatocellular carcinoma, and microsatellite instability (MSI)-high or mismatch repair gene (MMR)-deficient colorectal cancer (Table 1) [20–35]. It has been observed that pneumonitis may be associated with responses to PD antibodies [36, 37].

Nivolumab is being explored in more and more cancer types. Twenty patients with platinum-resistant ovarian cancer were treated with nivolumab in a phase II trial. Patients received up to six cycles (four doses per cycle). Twenty nivolumab-treated patients were evaluable at the time of the report and found to have ORR of 15%. Two of the responding patients had a durable CR (in the 3 mg/kg cohort). At the termination of the study, the median PFS was 3.5 months and the median overall survival (OS) was 20.0 months. The encouraging results from this pilot study of nivolumab in patients with platinum-resistant ovarian cancer suggest potential benefit of PD-1 antibody for refractory ovarian cancer [38]. Nivolumab is being studied in a phase I trial as a maintenance therapy for patients with high-risk hematological malignancies (NCT02985554). More than 350 trials of nivolumab have been registered on clinicaltrials.gov.

The article "Recent development in clinical applications of PD-1 and PD-L1 antibodies for cancer immunotherapy" was published in 2017. Journal: J Hematol Oncol.

Currently, pembrolizumab has FDA approved indications of seven different types of advanced malignancies. These malignancies include melanoma [39, 40], NSCLC [41–44], HNSCC, urothelial carcinoma, Hodgkin’s lymphoma [45], and gastric cancer [46, 47] (Table 1). Among these, FDA approved one indication for any malignancy with high microsatellite instability or mismatch repair gene (MMR) deficiency [48]. However, response to pembrolizumab in a gastric patient with stable MSI and proficient MMR has been observed [49]. Pembrolizumab has also been reported to be active in other highly refractory malignancies, such as Ewing’s sarcoma [50]. Recently, pembrolizumab was reported to be active in patients with refractory large cell lymphoma of the mediastinum [51].

Pembrolizumab has been studied in 26 patients with advanced Merkel cell carcinoma who had not received previous systemic therapy [52]. The overall response rate was 56%. The responses were seen in tumors with positive Merkel cell polyomavirus as well as in those with negative viral infections.

Atezolizumab is approved for treatment of advanced NSCLC and urothelial carcinoma [53–61]. The clinical activity of atezolizumab (MPDL3280A) in renal cell carcinoma (RCC) has been evaluated in 70 patients with metastatic RCC [62]. There were 63 with clear cell RCC and 7 with non-clear cell histology. These patients received atezolizumab every 3 weeks. PD-L1 expression was assessed with the Ventana SP142 assay on tumor cells and tumor-infiltrating immune cells (IC). For patients with clear cell RCC, the OS was 28.9 months (95% CI, 20.0 months to not reach) and PFS was 5.6 months (95% CI, 3.9 to 8.2 months). The ORR was 15% (95% CI, 7 to 26%). When the response was correlated with PD-L1 expression on IC cells, it was found that higher response rate was seen in PD-L1 expression ICs (18% RR in IC1/2/3, 9% RR in IC0). This study provided data to guide further trials with atezolizumab in RCC.

Durvalumab is approved for treatment of advanced urothelial carcinoma [63, 64]. Recently, the result of PACIFIC study was reported [65]. This was a randomized, placebo-controlled study of consolidation therapy for non-resectable stage III NSCLC after 2 cycles of planned chemoradiotherapy. Durvalumab was given as 10 mg/kg iv infusion over 30 min every 2 weeks up to 12 months. The PFS was significantly better for durvalumab (16.8 months, 95% CI 13 to 18.1 m) than that of the placebo arm (5.6 m, 95% CI, 4.6–7.8 m), *p* < 0.001). Overall survival as the secondary endpoint favored durvalumab, whereas the safety measures were similar in both groups. From this study, durvalumab was found to prolong PFS for approximately 11 months.

The article "Recent development in clinical applications of PD-1 and PD-L1 antibodies for cancer immunotherapy" was published in 2017. Journal: J Hematol Oncol.

Avelumab is approved for treatment of advanced Merkel cell cancer and advanced urothelial carcinoma [66, 67]. In a dose-escalation phase 1a trial, avelumab has demonstrated an acceptable safety profile and early suggestion of activity in patients with advanced solid tumors [68]. A phase Ib dose-expansion cohort of that trial was done in a cohort of patients with advanced, platinum-treated non-small-cell lung cancer (NSCLC) [69]. In this trial, 184 patients were treated with avelumab and followed for a median of 8.8 months. Severe adverse events (SAE) occurred in 44% of the 184 patients. The most common treatment-emerging adverse events (TEAE) among the 184 patients were fatigue 25%, infusion-related reaction (IRR) 21%, and nausea 13%. The ORR was 12% (95% CI 8–18), including 1 CR and 21 PR. In addition, 38% had stable disease. Further study on avelumab for advanced NSCLC appears to be warranted.

## Combination studies of PD-1 and PD-L1 antibodies with chemotherapy

In an attempt to enhance clinical benefits of cancer immunotherapy, PD antibodies are being evaluated in clinical trials in combination with chemotherapeutic agents [70]. The benefit of PD antibody in combination with radiation remains to be determined [71].

Nivolumab in combination with ipilimumab has been shown to improve progression-free survival of and approved for unresectable or metastatic melanoma [72]. A recent update from this trial revealed benefit on prolonged 3-year overall survival [73]. Nivolumab plus ipilimumab combination was studied in an open-label, phase 1, multi-cohort study (CheckMate 012) treatment-naïve patients with recurrent stage IIIb or stage IV NSCLC [74]. The first-line nivolumab plus ipilimumab was tolerable and showed a high response rate. This study supports further clinical trial of this combination in a phase 3 study.

Nivolumab plus platinum-based doublet chemotherapy (PT-DC) was evaluated for safety and tolerability as first-line therapy in 56 patients with advanced NSCLC [75]. Nivolumab plus PT-DC were given concurrently every 3 weeks for 4 cycles. This was followed by nivolumab alone as maintenance until progression or unacceptable toxicity. SAEs occurred in 45% of the patients. Seven percent had pneumonitis. AE-related discontinuation rate was reported more with the combination. Similar responses were seen in all dose levels irrelevant of PD-L1 expression. 2-year OS rate reached 62% in the nivolumab 5 mg/kg plus PT-DC group. This may warrant further investigation.

The article "Recent development in clinical applications of PD-1 and PD-L1 antibodies for cancer immunotherapy" was published in 2017. Journal: J Hematol Oncol.

Pembrolizumab was studied in combination with the doublet chemotherapy of carboplatin and pemetrexed in a multicenter randomized phase II study for patients with chemotherapy-naïve stage IIIB/IV non-squamous NSCLC and without EGFR or ALK mutations (KEYNOTE-021) [76]. In this study, PD-L1 tumor proportion score was stratified as < 1% vs >/= 1%. A total of 123 patients were enrolled in this published report. Among these patients, 60 received pembrolizumab plus chemotherapy (the combination group) and 63 had chemotherapy alone. Four cycles of pembrolizumab 200 mg plus carboplatin area under curve 5 mg/mL per min and pemetrexed 500 mg/m2 every 3 weeks were given to all patients. This was followed by pembrolizumab for 24 months and indefinite pemetrexed maintenance therapy versus indefinite pemetrexed maintenance therapy alone. At disease progression, those patients in the pemetrexed alone group were allowed for crossover to receive pembrolizumab. The primary endpoint was objective response rate (ORR). The ORR in the combination group was 55% (95% CI 42–68). This was significantly better than that in the pemetrexed alone group (29%; 18–41) (*p* = 0.0016). The incidence of severe treatment-emerging adverse events (TEAEs) was similar, and the most common ones were anemia and neutropenia. This was the first prospective randomized study that showed a benefit of a triplet regimen over doublet chemotherapy. This combination modality has been approved by FDA as the first line treatment for metastatic non-squamous NSCLC (Table 1). The benefit of adding pembrolizumab to platinum-doublet is being confirmed in two ongoing international, randomized, double-blind, phase 3 studies, KEYNOTE-189/NCT02578680 and KEYNOTE-407/NCT02775435.

## Combination studies of PD-1 and PD-L1 antibodies with other agents

Bevacizumab was combined with atezolizumab in a trial for metastatic RCC. When intra-tumoral CD8(+) T cells were enumerated and compared, it was found that the T cells increased in number following combination treatment. Biomarkers were examined in the study. Increase in chemokines was most notable for CX3CL1 (fractalkine) and its receptors. Following bevacizumab and atezolizumab combination treatment, more lymphocytes were seen in tumor tissues. This study suggests that the bevacizumab and atezolizumab combination improves antigen-specific T-cell migration [77].

Durvalumab was studied in a phase Ib trial in combination with osimertinib in NSCLC patients with EGFR activating mutations. The part A enrolled patients who were pretreated with EGFR tyrosine kinase inhibitors (TKI), and the part B enrolled treatment-naïve NSCLC patients. This combination was terminated for further enrollment due to high incidence of interstitial lung disease (38%) [78]. In a separate study, durvalumab was evaluated in a phase I trial in combination with gefitinib in treatment-naïve patients with NSCLC [79]. Early results appeared to be encouraging yet higher incidence of grade 3/4 liver enzyme elevation (40–70%) was observed. Atezolizumab was also studied in a phase I trial in combination with erlotinib in NSCLC patients with EGFR activating mutations [80]. In this report, 28 patients were included. TEAEs were seen in 50% of the patients, though no pneumonitis was reported. Early results from combination of EGFR TKIs with immunotherapy revealed higher incidence of TEAEs. Therefore, the combination therapy of EGFR TKI and immunotherapy remains investigational [78].

The article "Recent development in clinical applications of PD-1 and PD-L1 antibodies for cancer immunotherapy" was published in 2017. Journal: J Hematol Oncol.

PD-1 antibodies are also being studied in combination with indoximod, an inhibitor of indoleamine 2,3-dioxigenase 1 (IDO1) (NCT03301636) [81]. In a single arm phase 2 study of indoximod in combination with immunotherapy for patients with metastatic melanoma, a large majority of patients received indoximod with pembrolizumab as reported in an interim analysis [82]. Indoximod was given as 1200 mg PO twice daily concurrently with pembrolizumab (3 mg/kg q 21 days). The primary endpoint was ORR. In this report, 60 patients received the indoximod/pembrolizumab combination. The ORR was 52% (CR 8% + PR 44%). The combination was well tolerated. GI toxicities, anemia (17%), and hyperglycemia (17%) were the most common adverse events. A randomized phase 2/3 study of indoximod in combination with pembrolizumab or nivolumab is ongoing in patients with advanced melanoma (NLG2107, NCT03301636). Other IDO inhibitors are also being evaluated in combination with immunotherapy [81].

## Bioassays for PD-L1

The discovery of targetable oncogenes led to the routine molecular testing for gene mutations, such as those genes encoding epidermal growth factor receptor (*EGFR*) and *BRAF* V600E, *ALK*, the rat osteosarcoma (*ROS1*), *FLT3*, and *IDH*1/2 [41, 83]. More and more companion or complementary diagnostic assays are being approved upon approval of pharmaceutical products. A companion diagnostic assay is defined as a necessary test for the safe and efficacious use of a corresponding drug or biological product, whereas a complementary diagnostic assay is a test that evaluates a biomarker for the companion product to assess the risk/benefit ratio for a subset of patients [84, 85]. A complementary assay is not deemed essential in decision-making for the companion product. Avelumab was approved without a companion/complementary assay (Table 2).

The article "Recent development in clinical applications of PD-1 and PD-L1 antibodies for cancer immunotherapy" was published in 2017. Journal: J Hematol Oncol.

**Table 2:** Bioassays for PD-L1 expression

Antibodies	Bioassays
Pembrolizumab	Dako 22C3
Nivolumab	Dako 28-8
Atezolizumab	Ventana SP142
Durvalumab	Ventana SP263
Avelumab	NA

*NA* not applicable

Evaluation of PD expression on tumor cells and tumor-infiltrating T cells assists clinical decisions [86–88]. A variety of detection platforms were studied at different levels (protein, mRNA). Four immunohistochemistry (IHC)-based assays have been approved by FDA (Table 2). These assays include Dako 22C3, 28-8, and Ventana SP142 and SP263 [89, 90]. These bioassays have disparate positivity cut-off points and scoring systems in different tissue types. Therefore, standardization of clinical decision-making proves to be highly challenging.

Multiple studies have suggested that PD-L1 expression is affected by the specimen size, biopsy location, variable components of tumor and immune microenvironment, and tumor transformation [89]. To use PD-L1 as a predictive biomarker in clinical practice, these factors should be taken into consideration.

There exists a soluble form of PD-L1 (sPD-L1) in the sera of patients [91–94]. It remains unclear whether sPD-L1 level has correlation with clinical response to the checkpoint inhibitor treatment. It has been suggested that high sPD-L1 levels correlate with poor prognosis [95–98]. Liquid biopsy is increasingly used as a substitute of tissue sampling [99]. The value of liquid biopsy results and correlation with response to PD antibodies are uncertain at this time. Further development of multi-parameter biomarker panels is urgently needed.

## Conclusion and future directions

PD antibodies are revolutionizing cancer immunotherapy. The clinical use of PD antibodies is rapidly expanding. It has been shown that treatment history with hypomethylating agents appears to enhance response to PD-1 antibody [45]. Recent reports have shown that pembrolizumab is able to enhance CAR-T cell activity [100, 101]. Incorporation of PD antibodies into chemotherapy regimens is in active clinical investigations. Combination of PD antibodies with small molecule inhibitors such as IDO inhibitors and TKIs may further increase clinical efficacy.

## Abbreviations

HNSCC: Head and neck squamous cell carcinoma
NSCLC: Non-small cell lung cancer
PD: Programmed death
RCC: Renal cell carcinoma
UCC: Urothelial cell carcinoma
